This article has been retracted.

# Secure transmission for IoT wireless energy-carrying communication systems

**DOI:** 10.1371/journal.pone.0289251

**Published:** 2023-08-03

**Authors:** Pingxin Wang, Zhen Jing, Zhi Zhang, Qing Wang, Congcong Li, Hongxia Zhu

**Affiliations:** State Grid Shandong Electric Power Company Marketing Service Center (Measurement Center), Jinan, Shandong, China; Xidian University, CHINA

## Abstract

The wireless energy-carrying communication method for the Internet of Things (IoT) presents several difficulties for information security such as eavesdropping or data loss. To solve these issues, this paper presents a new secure transmission method for IoT wireless energy-carrying communication systems. In this method, first the secret message is turned into a word, delivered to the intended recipient and unlawful listener, respectively, and the received message is characterized as an entropy function. The message is iteratively solved using the block coordinate descent technique, and for each iteration, a digital baseband signal containing the receiver’s secret message symbol and the matching beamforming vector is delivered. By concurrently optimizing the transmit beamforming vector, the noise covariance matrix, and the receiver power allocation factor based on a design that complies with the security rate and energy acquisition limitations for each receiver, the overall system transmit power is reduced. The Lagrangian method is used to solve the secure transmission problem of the communication system based on an iterative block coordinate descent algorithm, as well as to change the nonconvex problem into a convex problem and precisely derive the upper and lower bounds of the original transmission problem. In comparison to the conventional policy transmission scheme, the experimental results demonstrate that the DIPS (Digital Image Processing System) scheme can increase the STP (Signaling Transfer Point) by approximately 34.16 percent in the eavesdropper independent eavesdropping and joint eavesdropping scenarios. The usefulness of the secure transmission strategy for wireless energy-carrying communication systems is confirmed by this investigation.

## 1. Introduction

Realizing the interconnectedness of things, the Internet of Things (IoT) is the real-time gathering and transmission of data via intelligent sensing devices [1–3]. IoT will have a significant influence on the growth of social productivity in the 21st century and is a "important productivity" that will fuel the fast expansion of the global economy in the future as a frontier of science and technology that has garnered considerable attention in the world today [4–6]. At the same time, artificial intelligence and technological advances in communication networks such as IoT, can play a vital role in improving the economy of natural resources [7]. IoT-based technologies can be useful in various fields such as Entrepreneurial Business [8], development of smart cities and sustainable planning of the urban environment [9], etc. Nevertheless, one of the basic requirements to achieve the goals outlined for IoT-based technologies in all its applications is to meet the security requirements such as the integrity of communications. In order to maintain the integrity of communication, two strategies have emerged in recent years: energy harvesting technology and increasing the energy effectiveness of communication networks [10]. The former is the rational allocation of limited resources with the help of some wireless communication techniques to reduce energy consumption, such as MIMO (fiber optic access), collaborative communication, and network coding techniques [11, 12]. The latter advocates the harvesting of renewable energy from the surrounding environment to power the nodes in the communication network, which not only captures energy but also these energies are renewable and sustainable. Compared to the former, it is clear that energy harvesting techniques not only improve the system spectrum utilization but also have the least negative impact on energy conservation and environment [13]. It is also the relatively safe, most economically efficient and suitable solution available.

Of course, there are various forms of energy harvesting, and the early energy harvesting is mainly to convert the natural wind, water, tidal energy, etc. into electricity. The current mainstream energy harvesting technology is to collect energy from RF signals in the surrounding environment, and then convert it into electrical energy for direct use or storage for future use. In fact, there are a large number of RF (electromagnetic signal) signals in the surrounding environment where people live, and these signals are stored in the air in the form of waves, which also carry information and energy. If the energy of the air "wave" is collected and used for power supply, it can greatly extend the working time of some energy-limited equipment and achieve the purpose of reducing the energy consumption of communication networks. Therefore, the wireless energy-carrying communication technology has received extensive attention and research since its introduction, and its development has a broad prospect and is one of the hot technologies for future communication [14].

The literature investigates a secure and reliable transmission method for a multi-cell, multi-user, large-scale multiple-input, multiple-output system with active eavesdroppers using multiple antennas [15]. Considered is a time-division duplex system where uplink training is necessary and an active eavesdropper may target the training period to contaminate the transmitter’s pilot. As a result, the downlink transmission phase’s precoding is forced to implicitly beamform in the direction of the listener. The best power allocation technique for the transmitted signal and generated noise is expressed in closed form for the scenario of a single antenna active eavesdropper, and the minimal transmit power necessary for dependable and secure communication is determined. According to the literature [16], UAVs may assist small cell base stations in traffic offloading through radio backhaul to enhance coverage and boost rates. Investigated is the safe transmission of scalable video on ultra-dense networks with the assistance of UAVs and caching. According to the suggested plan, UAVs might serve as SBSs (small cell base stations) and transmit video to mobile users over a number of small cells. The idle SBS may also be used to create jamming signals to prevent eavesdropping for secure communication. This scheme’s feasibility requirement is developed, and its secrecy effectiveness is assessed. For discrete cosine transform precoded orthogonal frequency division multiplexing visible light communication systems, a two-layer picture encryption technique is presented in the literature [17]. The transmitted picture is initially encrypted in the proposed technique using a chaotic scrambled sequence produced by a hybrid 4-D super and Arnold map in the top layer. In order to further increase the security of the transmitted picture, the encrypted image is next transformed into a digital QAM (quadrature amplitude) modulated signal and re-encrypted using a chaotic scrambling sequence based on the Arnold map in the physical layer. The results demonstrate that secure image-based transmission is accomplished by the suggested two-layer chaotic scrambling approach. According to the literature [18], the transmission should be meticulously planned to guarantee security and effectiveness in a multi-untrusted relay network. To enhance secure communication, a novel technique with symbol separation and beamforming is suggested. The segregated real and imaginary sections of the secret symbols are first sent through the top two relays with the highest channel gain. After that, the directional beamforming is carefully planned to optimize the reception of both actual and fictitious components by the two relay stations that have been chosen. With a high BER at the untrusted relay station and improved BER performance at the destination, the suggested approach offers full physical layer security.

Technological advances may affect natural resources. This destructive effect can be the result of creating environmental pollution or depletion of natural resources. Therefore, in various researches, the topic of technological innovations and environmental responsibility has been addressed. Research in [19] has focused on the natural gas supply for environmental sustainability under COP26 UN meeting and studied on the factors of technology, urbanization and economic complexity index in the top 15 natural gas supplier economies. In [20], a study was conducted about the affection of technology advancements on mental health. This research studies the destructive effect of internet addiction on mental health of university students. The research conducted in [21] studied the impact of interactive leadership on organizational creativity, which is possible through information sharing between the leader and the employees of the organization. In this regard, new communication technologies can play an effective role. The study [22], is an attempt to explore how business firms navigate employees’ technology-driven behavior and corporate social responsibility sustainable practices for tax avoidance to affect firms’ performance. This study shows that sustainable corporate social responsibility practices significantly moderate tax avoidance effect on business firms’ performance. In general, investing in renewable energy is one of the important factors in achieving sustainable energy sources, which is reachable through green technological innovations and has been studied in [23, 24]. Research in [23], studied the role of environmental tax, green finance and geopolitical risk in investment in renewable energy (IRE) sources. Also, research in [24] examines the impact of green technology innovation, financial development and green finance on green total factor productivity (GTFP) in China from 2011 to 2021. Research in [25], conducted a study about the link between ecology and health outcomes, accounting for the criticality of human capital and energy use in the middle east and north Africa countries.

The literature [26] takes into account secure downlink transmission in indoor multiple-input, single-output visible communication networks. To increase the feasible secrecy rate within the amplitude restrictions imposed by the constrained dynamic range of the light-emitting diode, the design of a transmit beamformer is examined. Consideration is given to the more likely scenario of faulty channel information on the connection between the receiver and the eavesdropper. The technique models the receiver channel uncertainty as a spherical set and attributes it to restricted feedback. However, if there is no input from the eavesdropper, the transmitter should use the line-of-sight channel gain equation to map the hypothetical position and direction of the eavesdropper as an estimate of the channel gain. The suggested secure file transmission method in the aforementioned literature has weak internal security safeguards and is susceptible to viral assaults during file transfer, which might lead to data loss or virus infection. Therefore, this paper constructs a secure transmission model for IoT, optimizes the power of the corresponding beamforming vector using block coordinate descent algorithm, locates the user confidential information encoding as an entropy function, and derives the secure transmission problem of the system by Lagrangian method. First, time-domain switching type energy-carrying communication network model is taken into consideration, which has multiple cells, multiple users, and multiple eavesdroppers. The transmitter dynamically shifts between energy transport and information transmission depending on the channel condition in order to fulfill the various needs for energy transport and information transmission, altering the conventional fixed allocation strategy for both. This makes it possible to thoroughly assess both the stability and efficiency of energy transmission as well as the dependability and security of information transfer under the conditions of both independent and combined eavesdropping by eavesdroppers. The impact of switching threshold on system performance is then investigated in order to strike a balance between system security and dependability. Next, a switching threshold optimization technique is created to increase secrecy throughput while staying within an energy budget. The resilience of secure transmission in the communication system is lastly supported by experimental data.

## 2. IoT secure transmission model

A sensor node is a small embedded device that typically consists of four basic components: data acquisition, data processing, wireless communication, and power supply. It uses wireless communication technology for data forwarding as well as self-organization for networking, giving it the dual functionality of data acquisition and data fusion. It is possible to more actively and effectively address the IoT data transmission security issue by actively building the privacy data security transmission model with the security during the privacy data transmission process as the research goal. The built-in IoT security transmission model is shown in Fig 1.

**Fig 1:** IOT secure transmission model.

As can be seen from Fig 1, the IoT secure transmission model consists of the ONS (Object Name Resolution Service) query mechanism for trusted anonymous authentication and the trusted anonymous transmission mechanism for item information. Among them, TAS (Vacuum Time Speed) generates the username of query system for L-ONS (Local Telephone Network System) in the registration stage, and generates temporary identity information for it to complete the authentication of identity legitimacy and platform trustworthiness for L-ONS. In the item information trusted anonymous transmission mechanism R-TIS (Reid Technology and Information Service) encrypts the query information layer by layer with the session keys of adjacent nodes from back to front in the order of each node in the response link. During transmission, the response data is decrypted in one layer for each passing node until the data is completely decrypted, and the intermediate nodes can verify the integrity of the forwarded data based on the signed encryption information of the precursor node and identify the authenticity of the forwarding path based on the routing information. During the data transmission process, the security during the data transmission process can be effectively guaranteed by the construction of the privacy data security transmission model, which is of great practical value.

## 3. Wireless portable collaborative communication technology

Today, communication networks have an undeniable role in accelerating the implementation of organizational processes and facilitating information transfer mechanisms. The importance of this was well proven in pandemic conditions of Covid-19 [27–29]; So that in most organizations, employees used different communication networks to do their work and after that, the scope of communication networks in organizations has always grown. In such a situation, the utilizing sustainable and secure strategies to improve the performance of communication networks is of great importance [30, 31], and in this section, efforts are made to meet this basic requirement. The framework of the proposed method is depicted in Fig 2. The remainder of this section is devoted to describing the steps of the proposed method.

**Fig 2:** Diagram of the proposed method.

### 3.1 Security rate definition

Consider a communication network that carries energy and has a number of resource centers, plenty of energy-constrained consumers, and passive listeners. The easiest of the three fundamental relay forwarding techniques to use is amplified forwarding. The relay node employing the AF (Amplified Forwarding) method does not parse the signal after receiving the information from the source node; instead, it amplifies and forwards the information directly to the target node using its own power, as well as amplifying and forwarding the relay receiving link’s noise. This will lead to a false code situation for the information received by the target node. However, because of the simple implementation process of the amplify-and-forward method and its low latency characteristics, which can effectively reduce the complexity of algorithm design and hardware cost, the AF method is widely used in collaborative communication systems with low transmission quality requirements and low latency.

The eavesdropping channel model commonly used in physical layer security research was proposed by Wyner. In this model, the legitimate sender Alice sends a confidential message that is first encoded into a code word, and the destination receiver Bob and the illegitimate eavesdropper Eve receive the confidential message sent by Alice, respectively. Specifically, the confidential message *w*^*k*^∈*W*^*k*^ sent by Alice is first encoded as code word *x*^*n*^. Then, the legitimate destination receiver Bob and the illegitimate eavesdropper Eve receive the message as *y*^*n*^ and *z*^*n*^, respectively. The suspicion rate *R*_*e*_ is defined as:

$$R_{e}=\frac{1}{n}h(w^{k}|z^{n}))$$ (1)

where $h(w^{k}|z^{n})$ is the entropy function, and $0\leq R_{e}\leq h(w^{k})/n$. When $R_{e}=h(w^{k})/n$, i.e., equivalent to $I(z^{n},w^{k})=0$, the amount of mutual information between *z*^*n*^ and *w*^*k*^ is zero at that time, it means that the illegal eavesdropper Bob does not receive any useful information, so the communication is absolutely secure. Here a concept of absolute security rate is defined, i.e., the amount of information that the sender sends to the destination receiver in absolute security when the $\left(2^{nR_{s}},n\right)$ encoding scheme is utilized.

The absolute safe rate *R*_*s*_ is reachable if for any *ε*,*ε*′>0 it is always possible to find a $\left(2^{nR_{s}},n\right)$-coded sequence that satisfies for any *n*≥*n*(*ε*,*ε*′):

$$P_{e}\leq \varepsilon^{\prime }$$ (2)

$$R_{s}-\varepsilon \leq R_{e}$$ (3)

where *P*_*e*_ represents the probability of error during message decoding and represents the reliability of message transmission. After giving the concepts of *R*_*e*_ and *R*_*s*_, the concept of safe capacity is further introduced. The system safety capacity *C*_*s*_ is the maximum value of the absolute safety rate.

When considering the multi-antenna eavesdropping channel scenario, both Alice, Bob, and Eve have multi-antenna scenarios. At this point, the achievable security rate of the MIMO eavesdropping channel can be defined as:

$$R_{s}={\left[\log\;\det(I_{N_{r}}+H_{d}Q_{x}H_{d}^{H})-\log\;\det(I_{N_{e}}+H_{e}Q_{x}H_{e}^{H})\right]}^{+}$$ (4)

where *Q*_*x*_ denotes the transmission covariance matrix of the input signal, the unit matrix of *Q*_*x*_ = *E*{*XX*^*H*^}, $I_{N_{r}}$ is the unit matrix of *N*_*r*_×*N*_*r*_, and *H*_*d*_ and *H*_*s*_ denote the wireless channels from Alice to Bob and Eve, respectively.

### 3.2 Block coordinate descent algorithm

The coordinate descent algorithm, which is an extension of the block coordinate descent technique, works on the premise that, for every optimization problem, whether it is solvable or not:

$$\min f(x)=f(x_{1},x_{2},\ldots ,x_{n})$$ (5)

$$s.t.x_{i}\in X_{i},i=1\ldots .,n$$ (6)

The optimization problem (5) can be solved iteratively according to the following Eq (6). Specifically, during each iteration, a set of optimization changes is first fixed, and then another set of variables is updated, alternating iterations until convergence. For example, in solving the optimal solution of the chunked coordinate vector *x*_*i*_ firstly, the remaining variables are regarded as constant values, and $x_{i}^{k+1}$ is obtained according to Eq (5) and finally:

$$x^{k+1}=(x_{1}^{k+1},\ldots x_{i}^{k+1},\ldots x_{n}^{k+1})$$ (7)

$$x_{i}^{k+1}=\arg\underset{x_{i}\in X_{i}}{\min}f(x_{1}^{k+1},\ldots x_{i-1}^{k+1},\ldots ,x_{i},x_{i+1}^{k},\ldots x_{n}^{k})$$ (8)

When sending covert communications, the sender often includes fake noise to obstruct prospective listeners and lessen their ability to eavesdrop on the conversation. The digital baseband signal transmitted may thus be represented as follows:

$$X=\sum_{k=1}^{K}w_{k}s_{k}+v$$ (9)

where *s*_*k*_ and $w_{k}\in {\mathbb{C}}^{N_{t}\times 1}$ represent the confidential message symbols and the corresponding beamforming vectors sent to the *k* rd receiver, respectively. $v\in {\mathbb{C}}^{N_{t}\times 1}$ represents the artificial noise vector, which obeys the distribution $v∼CN(0,V),V=vv^{H}\underline{≻}0$ and is the covariance matrix of *v*. For convenience, the indicator K={1,…,K} is defined as the set of all receivers, and $K_{-k}=\{1,\ldots ,k-1,k+1,\ldots K\}$ represents the set of all receivers except *k*. Assume $s_{k}∼CN(0,1),\forall k\in K$.

Assuming a power division receiver structure for each receiver, in particular, for *k* receiver ∀k∈K, $\rho_{k}(0\leq \rho_{k}\leq 1)$ part of the received power will be allocated to decode the message and the remaining 1−*ρ*_*k*_ to receive the acquired energy. Thus, the signal-to-dry ratio of the *k*th receiver after power division is expressed as follows:

$$\Gamma_{k}=\{\frac{\rho_{k}{\left|h_{k}w_{k}\right|}^{2}}{\rho_{k}(\sum j\neq k{\left|h_{k}w_{j}\right|}^{2}+Tr(h_{k}^{H}h_{k}V)+\sigma_{a,k}^{2})+\sigma_{s,k}^{2}}\}$$ (10)

where $h_{k}\in {\mathbb{C}}^{1\times N_{t}}$ represents the channel vector between the *k*nd sender and the receiver, $\sigma_{a,k}^{2}$ and $\sigma_{s,k}^{2}$ represent the antenna noise and the additional noise introduced by the signal processing for the *k*th receiver, respectively. On the other hand, the total harvest energy of the *k*th receiver is expressed as follows.

$$E_{k}=\eta_{k}(1-\rho_{k})(\sum_{j=1}^{K}{\left|h_{k}w_{j}\right|}^{2}+Tr(h_{k}^{H}h_{k}V))$$ (11)

where *η*_*k*_∈(0,1) denotes the received energy factor of the *k*nd receiver. The worst-case transmission scheme design is considered, where the potential eavesdropper decodes the message by using the continuous interference cancellation technique and all the acquired energy, so that the potential eavesdropper can eliminate all the multi-user interference. This secure transmission scheme design can be modeled as P1.

The Lagrangian method as well as the semidefinite relaxation method are used to deal with the problem of P1. The problem of P1 is first transformed into a more solvable form. Note ${\left|({\hat{h}}_{k}+\Delta h_{k})w_{k}\right|}^{2}$ This form is frequently applied in the problem of P1 by rewriting it as:

$$\begin{array}{l} {\left|({\hat{h}}_{k}+\Delta h_{k})w_{k}\right|}^{2}=w_{k}^{H}{\left({\hat{h}}_{k}+\Delta h_{k}\right)}^{H}({\hat{h}}_{k}+\Delta h_{k})w_{k}\\ \;=w_{k}^{H}({\hat{H}}_{k}+\Delta H_{k})w_{k} \end{array}$$ (12)

where ${\hat{H}}_{k}={\hat{h}}_{k}^{H}{\hat{h}}_{k}$ is the estimated constant covariance matrix of the channel state information.

Numerical simulations are used to verify and evaluate the security and robustness of the proposed transmission strategy. The parameters are set as *N*_*t*_ = 5, the number of receivers *K* = 3, the signal processing noise power $\sigma_{s,k}^{2}=-60dB$, the antenna noise power $\sigma_{a,k}^{2}=-50dB$ and $\gamma_{k}=\gamma_{o},\gamma_{e}^{m,k}=\gamma_{e}$ and $\xi_{k}=\zeta ,\forall k,$ $\eta_{k}=\eta =0.8,e_{k}=e_{0}$, and the large scale signal attenuation due to the distance between the sender and all receivers is 30 dB. Using the Rice channel model, the channel from the sender to each receiver is represented as follows:

$$h_{k}=\sqrt{\frac{K_{R}}{1+K_{R}}}h_{k}^{LOS}+\sqrt{\frac{1}{1+K_{R}}}h_{k}^{NLOS},\forall k$$ (13)

where $h_{k}^{LOS}\in {\mathbb{C}}^{N_{t}\times 1}$ and $h_{k}^{NLOS}\in {\mathbb{C}}^{N_{t}\times 1}$ denote the LOS deterministic part and Rayleigh decay deterministic part, respectively. *K*_*R*_ is the Rice factor, which is set to 5 dB. $h_{k}^{NLOS}$ each element obeys a mean of 0 and a variance of -30 dB.

In a secure cognitive wireless energy transmission system, the secondary link energy sender ET transmits the energy signal wirelessly to the energy receiver ER while the main transmitter delivers a private message to the principal user in the presence of a prohibited eavesdropper EA. They make use of the same spectrum assets. There are correspondingly and antennae set up for (PT), (PT), EA, ET, and ER. Energy transfer ET-generated co-channel interference is referred to as manufactured noise since it facilitates secure communication for the primary user. As a consequence, the main connection has the following safety rating:

$$R(Q,S)=R_{p}(Q,S)-R_{e}(Q,S)$$ (14)

where *R*_*p*_(*Q*,*S*) is the primary user reachable rate and *R*_*e*_(*Q*,*S*) is the eavesdropper reachable rate. *Q* and *S* are the covariance matrices of the main transmitter and energy transmitter transmissions. To design them separately, $H_{p}\in {\mathbb{C}}^{N_{p}\times N_{t}}$ denotes the channel matrices from the main transmitter to the main user and the eavesdropper, respectively.

The co-channel interference of the main transmitter may be seen as an energy source for the energy receiver. As a consequence, the energy receiver ER has gathered the following quantity of energy in total:

$$E(Q,S)=\eta (Tr(\left(G_{h}SG_{h}^{H}\right))+Tr(H_{h}QH_{h}^{H}))$$ (15)

where 0≤*η*≤1 represents the energy acquisition efficiency, $G_{h}\in {\mathbb{C}}^{N_{h}\times N_{s}}$ and $H_{h}\in {\mathbb{C}}^{N_{h}\times N_{s}}$ denote the channel matrices from the energy transmitter ET and the primary transmitter PT to the energy receiver ER, respectively. The energy transmitter ET provides energy signals to improve the main link’s safe transmission if the energy acquisition aim can be met. As a result, the primary goal of the design is to optimize the main link’s safety rate by maximizing the covariance matrix of the main transmitter’s PT and energy transmitter’s ET transmission, as well as to fulfill the energy receiver’s energy acquisition limitation. This may be mathematically represented by the following equation:

$$\underset{Q\underline{≻}0,S\underline{≻}0}{\max}R(Q,S)$$ (16)

$$s.tE(Q,S)\geq e_{o},Tr(Q)\leq p_{t},Tr(S)\leq p_{s}$$ (17)

where *e*_*o*_ is the minimum energy acquisition target value for the energy receiver. *p*_*t*_ and *p*_*s*_ denote the maximum transmitting power on the main transmitter PT and the energy transmitter ET, respectively.

The problem is transformed into an equivalent problem by using the BCD iterative algorithm. For this purpose, the aid of the Lemma is needed. Let *U*∈ℂ^*N*×*N*^ be an arbitrary matrix such as $U\underline{≻}0$. Consider the function f(W)=−Tr(WU)+log|W|+N, then:

$$-\log|U|=\underset{W\in {\mathbb{C}}^{N\times N},W\underline{≻}0}{\max}f(W)$$ (18)

where the optimal solution on the right side of the equation is W* = *U*^−1^.

## 4. Analysis of the safe transmission performance of wireless energy-carrying communication system

### 4.1 Convergence verification

Verify the convergence performance of the Lagrangian method. The convergence of the proposed algorithm for several randomly generated channels with a maximum transmit power of 1.2 W. The algorithm converges in only 2 to 3 iterations for different initial values. This is shown in Fig 3.

**Fig 3:** Convergence rate of the proposed algorithm update.

From Fig 3, the worst-case versus power is given for the channel cases with perfect and channel uncertainty ratios of $\sigma_{unc}^{2}=5\%$ and $\sigma_{unc}^{2}=10\%$, respectively. It is seen from the figure that the smaller the channel uncertainty ratio $\sigma_{unc}^{2}$, the smaller the performance loss for the same maximum transmit power, and the worst case is significantly reduced as the channel uncertainty ratio $\sigma_{unc}^{2}$ increases. This is because the higher the channel uncertainty, the more power is needed at the transmitter side to avoid eavesdroppers while satisfying the energy harvesting requirement, therefore, the higher the uncertainty the lower the security rate of the channel compared to the precision channel at the same maximum transmit power, and thus it will be lower.

By solving the problem, it is possible to obtain *Q*^*o*^ and *S*^*o*^. *ε*>0 represents the exact threshold value specified and *N*_max_ is the maximum value of the number of iterations. The cooperative precoding strategy for a secure wireless energy transfer scenario is examined in this work. As long as the secondary link’s energy acquisition requirements are met, the main link’s secure rate will be elevated. An iterative BCD-based method is used to handle the initial non-convex optimization problem. The secure transmission mechanism examined in this paper is shown to be effective in terms of secure rate and energy harvesting.

### 4.2 Validation of validity

By encoding user-confidential information into words using an IoT security transmission model, we demonstrate the efficacy of data security transmission in this paper’s wireless energy-carrying communication system. Wireless information transmission (WIT) must ensure that the transmitted information cannot be intercepted, whereas wireless energy transmission (WPT) only relies on RF signals to carry energy without ensuring its security. Wireless energy-carrying communication uses a wireless channel to carry both information transmission and energy transmission, but the security requirements of the two are different. By period splitting, the wireless energy-carrying communication technology makes it possible to transmit energy and information simultaneously. The downlink period Tdl (terminal display language) is divided into two intervals by the transmitter in the conventional scheme, but in reality, the wireless channel is random, so the conventional scheme is unable to dynamically adjust the time slot in accordance with the channel quality to satisfy the various requirements of reliable and secure energy and information transmission. In this study, numerical analysis and simulation using the Lagrangian approach are used to verify the effectiveness of the suggested transmission strategy. The energy conversion relationship is depicted in Fig 4 under the presumption that the channel fading coefficient, period, transmit power of all RCs (remote controls), number of antennas, users served, target rate and target security rate, and density are circuit parameters in NLM (news mailing list).

**Fig 4:** Non-linear/linear energy conversion curve.

The conversion efficiency of the NLM dynamically fluctuates with input power and is maintained in a very low range when the input power is low, leading to inefficient usage of the bulk of the energy, as shown in Fig 4. Energy resources benefit greatly from the fact that the effect of increased input power on boosting energy gain becomes more confined and shifts to a falling trend. When the output hits the saturation zone and the input power exceeds a specified range, this happens. The continuous dynamic is less concerning than this dynamic. In the context of "green communication," we utilize route loss as the WPT efficiency index and take into consideration its effect on energy efficiency in this article.

### 4.3 Transmission performance verification

The complementary probability curves of both CCOP (password proceeding buffer) and CSOP (administrator) are provided together with the definition of STP for a more understandable comparison study. Fig 5 shows how switching threshold affects WIT performance.

**Fig 5:** Effect of switching threshold on information transmission performance. (a) Effect of switching threshold on CCOP/CSOP/ITP, (b) Effect of switching threshold on STP/ITP.

Fig 5(A) illustrates how the development patterns of CCOP and CSOP are consistent with the findings of the COP and SOP (operating procedure) studies. This is because raising the switching threshold improves WIT’s average channel quality and information delivery (including reliability and security). The switching threshold, however, limits the potential for WIT. According to the definition of STP, Fig 5(B) shows that ASR and ITD (information technology) both have an effect on STP simultaneously. STP displays a non-monotonic shift with the change in switching threshold, however, since there is a game-like interaction between switching threshold and ASR and ITD. STP increases first, then decreases, since there is an optimal switching threshold that allows it to reach its maximum value. Moreover, it is shown that when the eavesdroppers eavesdrop jointly, the available STP considerably decreases even while the switching threshold at the greatest STP significantly increases. This is due to the fact that a higher channel quality is needed to permit secure transmission the more eavesdropping is a threat that must be avoided, resulting in the finest ASR and ITD balance feasible.

The higher the density of eavesdroppers, the greater the threat posed, and the higher the requirement for channel resources to ensure information security, so when the constraints are sufficiently loose, the optimal switching threshold increases with the increase in eavesdropper density, which includes 2 cases of independent eavesdropping and joint eavesdropping. With the tightening of the constraints, it is necessary to meet the requirements of the indicators at the cost of a certain performance loss. The relationship between the optimal switching threshold and the density of eavesdroppers is shown in Fig 6.

**Fig 6:** Relationship between optimal switching threshold value and eavesdropper density.

As can be seen from Fig 6, the minimum switching thresholds corresponding to the constraints are -3.37dB, -3.66dB, -5.08dB, -4.31dB (independent eavesdropping) and 0.08dB (joint eavesdropping). Therefore, for the scenario of independent eavesdropping, the EUR constraint is the strongest, and because the optimal threshold under the loose constraint always fails to meet the minimum requirement, the final switching threshold is the lowest threshold corresponding to the constraint -3.37 dB. While for the scenario of joint eavesdropping, the SOP constraint is the strongest, and the threshold under the loose constraint fails to meet the requirement when the density of eavesdroppers is low. The tighter the single constraint affects the value of the final switching threshold, the tighter the single constraint, the greater the gap between the final threshold and the optimal threshold under the loose constraint, and the more STP is lost.

The relationship between the STP and eavesdropper density can be reached under the 2 scenarios of independent eavesdropping and joint eavesdropping is shown in Fig 7.

**Fig 7:** Confidential throughput under different eavesdropper density conditions.

Fig 7 shows that the numerical findings and simulation results agree, demonstrating the accuracy of the derivation procedure. Additionally, the DIPS transmission strategy, when compared to the conventional policy beam transmission scheme, may successfully raise system average STP while maintaining energy limitations in both joint and eavesdropper independent eavesdropping situations. Whereas the DIPS scheme offers a greater level of security against eavesdropper-independent eavesdropping and gradually declines as eavesdropper density rises, this is due to the fact that as eavesdroppers become more advanced (in terms of capability or density), it becomes harder to thwart their eavesdropping. Additionally, the loss of STP due to SOP restrictions is especially apparent in the joint eavesdropping situation when the number of listeners is minimal. The DIPS method may still raise the STP by roughly 34.16 percent, as the graphic illustrates. Additionally, the feasible STP of the conventional policy scheme is severely constrained when the eavesdropper density reaches a certain point, and the system can scarcely interact securely, whereas the STP of the DIPS scheme may still be maintained at a certain level. In conclusion, the plan outlined in this article may significantly increase the security and dependability of information transfer.

### 4.4. Differential analysis verification

In order to study the performance of the proposed method more precisely, and verify the superiority of the proposed method, the difference between the observed values and the actual values has been evaluated using Root Mean Squared Error (RMSE), Mean Absolute Error (MAE) and Relative Error (RE) criteria. The RMSE criterion, shows the root of average squared difference between the observed and the actual values and can be calculated as follows:

$$RMSE=\sqrt{\frac{1}{N}\sum_{i=1}^{N}{\left({\hat{y}}_{i}-y_{i}\right)}^{2}}$$ (19)

Where, ${\hat{y}}_{i}$ represents the i-th observed data and *y*_*i*_ represents the corresponding actual value. Also, *N* represents the number of samples. On the other hand, the MAE criterion describes the average absolute difference between the observed and the actual values. This criterion is effective in more clear reflection of system error and can be formulated as follows:

$$MAE=\frac{1}{N}\sum_{i=1}^{N}\left|{\hat{y}}_{i}-y_{i}\right|$$ (20)

Finally, the RE criterion indicates the rate of difference between the observed and the actual values, which is calculated by dividing the difference between the observed values and the actual values by the actual values:

$$RE=\frac{1}{N}\sum_{i=1}^{N}\frac{\left|{\hat{y}}_{i}-y_{i}\right|}{y_{i}}$$ (21)

In Fig 8, the efficiency of the proposed method has been evaluated in terms of the mentioned criteria and the results have been compared with GA-LM-BP, LM-BP and BP methods in [32].

**Fig 8:** The efficiency of the proposed method in terms of RMSE, MAE and RE.

As shown in Fig 8, the proposed method outperforms compared methods in terms of RMSE, MAE and RE. According to these results, the proposed method obtains the RMSE of 0.0082; while the GA-LM-BP -as the closest method- produces RMSE value of 0.011. This means the proposed method can reduce RMSE by at least 25.45%. Also, the MAE of the proposed method is 0.008 which shows at least 27.27% reduction compared to the closest performing method. Finally, the proposed method reports 0.0108 for the RE criterion which means at least 22.86% reduction compared to other methods. These results, confirm the efficiency of the proposed method in transferring messages with lowest error rates and proves its performance in conserving the integrity of communication networks.

## 5. Conclusion

In the case that IoT wireless sensor nodes are unable to use encryption methods, a secure transmission model of privacy data that is actively developed to explore the security during the transmission of privacy data may deal with the security of IoT data transmission more actively and effectively. This study presents an opportunity secure transmission method for a time-domain switching type portable communication system. Simulation is utilized to demonstrate the effectiveness of the suggested strategy. The results are shown as follows:

- The NLM’s conversion efficiency, which varies dynamically with input power, corresponds to the minimum switching thresholds of -3.37 dB, -3.66 dB, -5.08 dB, -4.31 dB, and 0.08 dB. The dynamic information energy switching transmission scheme of the threshold is proposed, and the best performance of energy transmission and information transmission is carefully examined, taking into account the differential security requirements for energy transmission and information transmission as well as the time-varying characteristics of the wireless channel.
- The DIPS approach can effectively raise the system average STP while keeping the energy constraint in both the eavesdropper independent eavesdropping and collaborative eavesdropping scenarios. Even when there are few eavesdroppers present, the DIPS approach may still increase the STP by around 34.16 percent. It is shown how effective the proposed strategy is.
- The differential analysis results showed that the proposed method can reduce the RMSE, MAE and RE criteria, by at least 25.45%, 27.27% and 22.86%, respectively. Thus, the proposed method is an effective approach in transferring messages with lowest error rates and leads to conserving the integrity of communication networks.

The results of this research showed that the proposed method is an efficient strategy for secure transmission in IoT wireless energy-carrying communication systems and can be useful in real-world practical scenarios.

## Supporting information

S1 Data (XLSX)
